# An Improved Estimation for Heterogeneous Datasets with Lower Detection Limits regarding Environmental Health

**DOI:** 10.1155/2022/4414582

**Published:** 2022-07-12

**Authors:** Navid Feroze, Ali Akgul, Taghreed M. Jawa, Neveen Sayed-Ahmed, Rashid Ali

**Affiliations:** ^1^Department of Statistics, The University of Azad Jammu and Kashmir, Muzaffarabad, Pakistan; ^2^Department of Mathematics, Siirt University, Art and Science Faculty, 56100 Siirt, Turkey; ^3^Department of Mathematics, College of Science, Taif University, Taif 21944, Saudi Arabia; ^4^School of Mathematics and Statistics, Central South University, Changsha, 410083 Hunan, China

## Abstract

Analysis of environmental data with lower detection limits (LDL) using mixture models has recently gained importance. However, only a particular type of mixture models under classical estimation methods have been used in the literature. We have proposed the Bayesian analysis for the said data using mixture models. In addition, an optimal mixture distribution to model such data has been explored. The sensitivity of the proposed estimators with respect to LDL, model parameters, hyperparameters, mixing weights, loss functions, sample size, and Bayesian estimation methods has also been proposed. The optimal number of components for the mixture has also been explored. As a practical example, we analyzed two environmental datasets involving LDL. We also compared the proposed estimators with existing estimators, based on different goodness of fit criteria. The results under the proposed estimators were more convincing as compared to those using existing estimators.

## 1. Introduction

The environmental studies often encounter the exposure measurements falling below the LDL. These nondetectable observations are considered left censored observations [1, 2]. Hughes [3] discussed that the difficulty in modeling the environmental concentration datasets arises when some of the measurements are below the LDL. As the proportion of censored observations may not be trivial, failure to adjust the censoring in the analysis can produce seriously biased results with inflated variances. The most convenient method to adjust the censoring is to replace the censored observation by the detection limit. However, statistical properties of such methods are obscured. As an improvement, Paxton et al. [4] proposed the iterative imputation technique to settle the censoring issue, but this method did not consider the correlated structure of the data and parametric estimates.

Some authors have proposed the standard statistical distributions to model the left censored datasets. For example, Mitra and Kundu [5] used generalized exponential distribution, Bhaumik et al. [6] employed normal distribution, Leith et al. [7] and Jin et al. [8] used log-normal distribution, and Asgharzadeh et al. [9] considered Weibull model to model the left censored data from different situations. However, varying modeling capabilities of these models to model the left censored data has been reported by Vizard et al. [10]. Further, Moulton and Halsey [11] raised several concerns over using a standard statistical model to deal with such data. They argued that these datasets may be highly skewed to make most of the standard models inappropriate for analysis. Further, there may exist an additional subpopulation of the observations falling below the detection limit making the data heterogeneous or multimodal. Following these arguments, Moulton and Halsey [11] suggested the use of gamma mixture model (in their case) to model the left censored HIV RNA dataset. Taylor et al. [12] also emphasized that in case of larger proportion of nondetectable observations, a suitable model for analysis should be explored. They proposed log-normal mixture distribution to model the datasets with LDL. Some other authors including Moulton et al. [13] and Chen et al. [14] have suggested the use of mixture models for analyzing left censored data, especially when the proportion of censoring and skewness is high in the data. The use of mixture models also allows additional variability in the distributional shape as compared to some standard models. A recent article by Feroze and Aslam [15] considered the analysis of left censored mixture of the Weibull model.

Furthermore, most of the authors employing mixture models for analyzing left censored datasets have proposed maximum likely estimation (MLE) to estimate the model parameters. But, as the mixing cause missing data, MLE is often not suitable in estimating mixture models [16]. Following this argument, Hughes [3] proposed EM algorithm assuming normal mixture model to adjust the censoring issue in MLE. But the EM algorithm can also fail when the censoring rate is high [17]. These issues in the estimation of mixture models can be handled using a Bayesian approach. With informative priors, Bayesian estimation (BE) can produce significant gains in efficiencies of the estimates as compared to classical methods [18, 19]. The Bayesian estimators (BEs) can be biased but often have smaller mean squared errors (as compared to MLEs) and include additional prior information [20]. These methods are also applicable when the parameter estimates are correlated [21]. However, the Bayesian inference has not yet replaced the classical methods to model the heterogeneous environmental concentration datasets with LDL [22].

The generalized exponential (GE) distribution is very important distribution to model censored datasets. Recently, Gupta and Kundu [23] and Mitra and Kundu [5] identified that this model can be an appealing alternative to many standard models, such as gamma, Weibull, lognormal, log-gamma, exponential, and Rayleigh, to analyze the censored datasets. The mixture of GE models for analyzing the censored datasets has been more recently introduced. Teng and Zhang [24] proposed the estimation of model parameters from two-component mixture of GE models (2CMGEM) via EM algorithm. Ali et al. [25] discussed the application of 2CMGEM in modeling right censored data. Mahmoud et al. [26] considered 2CMGEM for obtaining predictions from the censored data. Wang et al. [27] discussed the applicability of 2CMGEM in medical sciences. Similarly, Kazmi and Aslam [28] advocated the employment of GE mixture model to fit various right censored datasets. More recent contributions regarding the analysis of 2CMGEM can be seen from the following works. Aslam and Feroze [29] considered the analysis of 2CMGEM under progressive censoring. Kluppelberg and Seifert [30] reported some important results from the conditional distributions of 2CMGEM. Yang et al. [31] discussed important inferences about 2CMGEM. Various properties of 2CMGEM were investigated. Hence, 2CMGEM is a very relevant model to analyze the censored dataset with mixture or heterogeneous behavior.

We have explored the advantages of Bayesian methods in modeling the heterogeneous environmental concentration data with LDL. First, we have employed the Bayesian mixture model approach using simulated datasets. As discussed by Momoli et al. [22], these datasets represent the real data from environmental studies and provide convenience by avoiding issues with empirical comparisons. Further, to investigate the advantages of the proposed methodology in real world, two real datasets regarding environmental concentrations with LDL have been used for the analysis. The 2CMGEM has been used as candidate model to analyze the mixture behavior of these datasets. The comparison of the proposed model with other mixture models, available in the literature to analyze the datasets with LDL, has been made. The comparison among different estimation methods has been discussed. Some advantages of using the proposed methodologies have been observed.

The remaining paper has been organized as follows.  Section 2 contains the estimation of model parameters using different estimation methods. In Section 3, the simulated datasets are considered for comparison of proposed estimators. In Section 4, two real examples have been used to discuss the applicability and suitability of the proposed estimators. The findings of the study have been reported in Section 5.

## 2. Material and Methods

This section contains the analytical estimation of model parameters under expectation-maximization (EM) algorithm, Lindley's approximation (LA), and Markov chain Monte Carlo (MCMC) method. In case of BE, the squared error loss function (SELF) and entropy loss function (ELF) along with an informative prior have been assumed for the estimation.

### 2.1. The Likelihood Function for 2CMGEM under Heterogeneous Data with LDL

The 2CMGEM has following probability density function:

(1) $$\begin{array}{c} f\left(x;\Omega \right)=\overset{2}{\underset{u=1}{\sum }}\pi_{u}\lambda_{u}\theta_{u}{\left\{1-\exp\left(-\theta_{u}x\right)\right\}}^{\lambda_{u}-1}e^{-\theta_{u}x}0<x<\infty , \end{array}$$

where **Ω** = (*λ*_1_, *θ*_1_, *λ*_2_, *θ*_2_, *π*_1_) is a parametric set and *λ*_*u*_, *θ*_*u*_ > 0, 0 < *π*_1_ < 1*u* = 1, 2.

The cumulative distribution function (CDF) for the 2CMGEM is

(2) $$\begin{array}{c} F\left(x;\Omega \right)=\overset{2}{\underset{u=1}{\sum }}\pi_{u}{\left\{1-\exp\left(-\theta_{u}x\right)\right\}}^{\lambda_{u}}0<x<\infty . \end{array}$$

Suppose, we generate a sample of size ‘*n*' from 2CMGEM. Further, suppose *n*_1_ = *nπ*_1_ and *n*_2_ = *n*(1 − *π*_1_) observations are generated from first and second components of the mixture, respectively. Let *X*_*k*+1_, ⋯, *X*_*n*_ are the largest *n* − *k*  observations about which we have complete information and remaining smallest ‘*k*' observations fall below the predetermined LDL. Since we have incomplete information regarding smallest ‘*k*' observations, they as assumed as censored. Hence, *x*_1(*k*_1_ + 1)_, ⋯, *x*_1*n*_1__ and *x*_2(*k*_2_ + 1)_, ⋯, *x*_2*n*_2__ are the observations with complete information from first and second component of the mixture, respectively. So, *k*_1_ and *k*_2_ are the starting observations censored from each component, respectively. Further, *m*_1_ = *n*_1_ − *k*_1_ − 1 and *m*_2_ = *n*_2_ − *k*_2_ − 1 are observed items (with complete information) from the first and second components of mixture, respectively, where *x*_*k*_ = min(*x*_1(*k*_1_ + 1)_, *x*_2(*k*_2_ + 1)_), *n* = *n*_1_ + *n*_2_, *k* = *k*_1_ + *k*_2_, and *n* − *k* = *m*_1_ + *m*_2_. The likelihood function for such heterogeneous dataset *x* = {(*x*_1(*k*_1_ + 1)_, ⋯, *x*_1*n*_1__), (*x*_2(*k*_2_ + 1)_, ⋯, *x*_2*n*_2__)} with LDL can be written as

(3) $$\begin{array}{c} L\left(\Omega \left|x\right.\right)\propto {\left\{\pi_{1}F_{1}\left(x_{k+1}\right)\right\}}^{k_{1}}{\left\{\left(1-\pi_{1}\right)F_{2}\left(x_{k+1}\right)\right\}}^{k_{2}}\left\{\overset{n_{1}}{\underset{i=k_{1}+1}{\prod }}\pi_{1}f_{1}\left(x_{1i}\right)\right\}\left\{\overset{n_{2}}{\underset{i=k_{2}+1}{\prod }}\left(1-\pi_{1}\right)f_{2}\left(x_{2i}\right)\right\}, \end{array}$$

where **Ω** = (*λ*_1_, *θ*_1_, *λ*_2_, *θ*_2_, *π*_1_). Putting the corresponding entries, we have the following.

The likelihood function for the heterogeneous dataset with LDL using 2CMGEM is

(4) $$\begin{array}{c} \begin{array}{c} L\left(\Omega \left|x\right.\right)=\pi_{1}^{k_{1}+m_{1}}{\left(1-\pi_{1}\right)}^{k_{2}+m_{2}}\overset{2}{\underset{u=1}{\prod }}\lambda_{u}^{m_{u}}\exp\left\{\left(\lambda_{u}-1\right)\overset{n_{u}}{\underset{i=k_{u}+1}{\sum }}\log\left(1-\exp\left(-\theta_{u}x_{ui}\right)\right)\right\}\\ \times \theta_{u}^{m_{u}}\exp\left(-\theta_{u}\overset{n_{1}}{\underset{i=k_{1}+1}{\sum }}x_{1i}\right){\left(1-\exp\left(-\theta_{u}x_{k+1}\right)\right)}^{\lambda_{u}k_{u}}, \end{array} \end{array}$$

### 2.2. Expectation-Maximization (EM) Algorithm

In case of missing observations, the EM algorithm can be used obtain the MLEs for the model parameters. We have used the EM algorithm similar to that proposed by Ruhi et al. [32]. LetΘ = (*λ*_1_, *λ*_2_, *θ*_1_, *θ*_2_) be the model parameters and *π*_1_ the mixing parameter for the 2CMGEM *f*_*r*_(*x*) where *r* = 1, 2.

Let us denote the observed random sample from 2CMGEM by *x*_*o*_ = (*x*_1_, ⋯,*x*_*n*_)′. Further, we assume the missing data vectors as *x*_*c*_ = (*y*_1_′, ⋯,*y*_*n*_′)′, where *y*_*j*_ is a 2-dimensional indicator vector containing zero-one observation and *y*_*jr*_ is one if the *x*_*j*_ is from *r*^th^ component of the mixture and zero elsewhere (*j* = 1, 2, ⋯, *n*; *r* = 1, 2). The complete dataset can be defined as *x* = (*x*_*o*_′, *x*_*c*_′). The iterations in any EM algorithm contain two steps. The conditional expectation of the complete data log-likelihood for the model parameters is computed in the first step called *E*-step. The *E*-step at (*z* + 1)th iteration is

(5) $$\begin{array}{c} I\left(\Omega ,\Omega^{\left(z\right)}\right)=\overset{n}{\underset{j=1}{\sum }}\overset{2}{\underset{r=1}{\sum }}{Ε}_{\Omega^{\left(z\right)}}\left(Y_{jr}\left|x_{o}\right.\right)\partial_{j}\ln\left\{\pi_{r}^{\left(z\right)}f_{r}\left(x_{j}\left|\Theta_{r}^{\left(z\right)}\right.\right)\right\}+\overset{n}{\underset{j=1}{\sum }}\overset{2}{\underset{r=1}{\sum }}{Ε}_{\Omega^{\left(z\right)}}\left(Y_{jr}\left|x_{o}\right.\right)\left(1-\partial_{j}\right)\ln\left\{\pi_{r}^{\left(z\right)}R_{r}\left(x_{j}\left|\Theta_{r}^{\left(z\right)}\right.\right)\right\}, \end{array}$$

where *R*_*r*_(*x*_*j*_|Θ_*r*_^(*z*)^) is a reliability function for the *r*^th^ component of the mixture. As (5) is linear in*y*_*jr*_, the *E*-step is implemented by taking the conditional expectation of *Y*_*jr*_ given the observed data *x*_*o*_, where *y*_*jr*_ denotes the observations of *Y*_*jr*_. Now, *Ε*_**Ω**^(*z*)^_(*Y*_*jr*_|*x*_*o*_) = *y*_*jr*_^(*z*)^. Using Bayes theorem, the posterior probabilities *y*_*jr*_^(*z*)^ are presented as

(6) $$\begin{array}{c} y_{jr}^{\left(z\right)}=\frac{\pi_{r}^{\left(z\right)}\left\{\partial_{j}f_{r}\left(x_{j}\left|\Theta_{r}^{\left(z\right)}\right.\right)+\left(1-\partial_{j}\right)R_{r}\left(x_{j}\left|\Theta_{r}^{\left(z\right)}\right.\right)\right\}}{\sum_{k=1}^{z}\pi_{r}^{\left(z\right)}\left\{\partial_{j}f_{r}\left(x_{j}\left|\Theta_{r}^{\left(z\right)}\right.\right)+\left(1-\partial_{j}\right)R_{r}\left(x_{j}\left|\Theta_{r}^{\left(z\right)}\right.\right)\right\}}. \end{array}$$

Next, the *M*-step is carried out. In this step, (5) is maximized with respect parameters of the model to estimate **Ω**^(*z* + 1)^. Since expressions containing *π*_*r*_ and Θ_*r*_ are not related, they can be maximized independently. We introduce the Lagrange multiplier Δ, with condition ∑_*r*=1_^2^*π*_*r*_ = 1., to obtain the expression for *π*_*r*_. The differentiation of (5) with respect to *π*_*r*_ is placed equal to zero as

(7) $$\begin{array}{c} \overset{n}{\underset{j=1}{\sum }}\frac{1}{\pi_{r}}y_{jr}^{\left(z\right)}+\Delta =0. \end{array}$$

The sum of (7) over *r* and with∑_*k*=1_^*z*^*y*_*jr*_^(*z*)^ = 1, and Δ = −*n* gives

(8) $$\begin{array}{c} \pi_{r}^{\left(z+1\right)}=\frac{1}{n}\overset{n}{\underset{j=1}{\sum }}y_{jr}^{\left(z\right)}. \end{array}$$

The MLES for Θ_*r*_ = (*λ*_*r*_, *θ*_*r*_), *r* = 1, 2 are obtained using iterative procedures. Both *E*-step and *M*-step are iterated for achieving the desired accuracy.

The steps to estimate the parameters of 2CMGEM using EM algorithm are as follows:.

- Step-1:determine the initial guess for parameters as *π*_1_^(0)^, *θ*_*r*_^(0)^, and *λ*_*r*_^(0)^ at *r* = 1, 2
- Step-2:using Step-1 compute the conditional expectation *y*_*jr*_^(*z*)^ for z^th^ iteration from (6)
- Step-3: for *z*^th^ iteration, derive MLE of *π*_1_^(*z* + 1)^ from (8) and MLEs of *θ*_*r*_^(*z* + 1)^ and *λ*_*r*_^(*z* + 1)^ using numerical procedures
- Step-4: replicate Step-2 and Step-3 to reach the desired convergence

### 2.3. Bayesian Estimation

The beta prior for parameter *π*_1_ and independent gamma priors for parameters *λ*_1_, *λ*_2_, *θ*_1_, *θ*_2_ have been assumed as

(9) $$\begin{array}{c} h\left(\pi_{1}\right)\propto \pi_{1}^{\mu_{1}-1}{\left(1-\pi_{1}\right)}^{\tau_{1}-1},0<\pi_{1}<1, \end{array}$$

(10) $$\begin{array}{c} h\left(\lambda_{u}\right)\propto \overset{2}{\underset{u=1}{\prod }}\lambda_{u}^{\mu_{2u}-1}\exp\left(-\tau_{2u}\lambda_{u}\right),\lambda_{u}>0, \end{array}$$

(11) $$\begin{array}{c} h\left(\theta_{u}\right)\propto \overset{2}{\underset{u=1}{\prod }}\theta_{u}^{\mu_{3u}-1}\exp\left(-\tau_{3u}\theta_{u}\right),\theta_{u}>0, \end{array}$$

where *μ*_1_, *τ*_1_, *μ*_2*u*_, *τ*_2*u*_, *μ*_3*u*_, *τ*_3*u*_ > 0, *u* = 1, 2 are the hyperparameters.

Under the assumption of independence, the joint prior density from (9)–(11), for the parametric set **Ω** = (*λ*_1_, *λ*_2_, *θ*_1_, *θ*_2_, *π*_1_) can be given as

(12) $$\begin{array}{c} h\left(\Omega \right)\propto \pi_{1}^{\mu_{1}-1}{\left(1-\pi_{1}\right)}^{\tau_{1}-1}\overset{2}{\underset{u=1}{\prod }}\lambda_{u}^{\mu_{2u}-1}\exp\left(-\tau_{2u}\lambda_{u}\right)\theta_{u}^{\mu_{3u}-1}\exp\left(-\tau_{3u}\theta_{u}\right),0<\pi_{1}<1,\lambda_{u},\beta_{u}>0. \end{array}$$

The general form of posterior distribution for the model parameters, combining (4) and (11), is

(13) $$\begin{array}{c} g\left(\Omega \left|x\right.\right)\propto L\left(\Omega \left|x\right.\right)h\left(\Omega \right). \end{array}$$

From (13), the posterior distribution for the parameters of 2CMGEM is

(14) $$\begin{array}{c} \begin{array}{c} g\left(\Omega \left|x\right.\right)\propto \pi_{1}^{k_{1}+m_{1}+\mu_{1}-1}{\left(1-\pi_{1}\right)}^{k_{2}+m_{2}+\tau_{1}-1}\overset{2}{\underset{u=1}{\prod }}\lambda_{u}^{m_{u}+\mu_{2u}-1}\exp\left\{-\tau_{2u}\lambda_{u}+\left(\lambda_{u}-1\right)\overset{n_{u}}{\underset{i=k_{u}+1}{\sum }}\log\left(1-\exp\left(-\theta_{u}x_{ui}\right)\right)\right\}\\ \times \theta_{u}^{m_{u}+\mu_{3u}-1}\exp\left\{-\theta_{u}\left(\tau_{3u}+\overset{n_{u}}{\underset{i=k_{u}+1}{\sum }}x_{ui}\right)\right\}{\left(1-\exp\left(-\theta_{u}x_{k+1}\right)\right)}^{\lambda_{u}k_{u}}. \end{array} \end{array}$$

We have used SELF and ELF for derivation of BEs. The BE under SELF is ${\hat{\Omega }}_{S}=Ε\left(\Omega \left|x\right.\right)$. On the other hand, the BE under ELF is ${\hat{\Omega }}_{E}={\left[Ε\left(\Omega^{-1}\left|x\right.\right)\right]}^{-1}$. Since the closed form expressions for BEs under the said loss functions are not available, the approximate BE methods have been used to compute the numerical results.

#### 2.3.1. Lindley's Approximation (LA)

In this section, the LA has been proposed for the approximate BE for parameters of 2CMGEM. For sufficiently large sample size, Lindley [33] proposed that a ratio of integrals have the form

(15) $$\begin{array}{c} I\left(\Omega \right)=Ε\left[W\left(\Omega \right)\right]=\frac{\int_{\Omega }W\left(\Omega \right)\exp\left\{K\left(\Omega \left|x\right.\right)+H\left(\Omega \right)\right\}d\Omega }{\int_{\Omega }\exp\left\{K\left(\Omega \left|x\right.\right)+H\left(\Omega \right)\right\}d\Omega }, \end{array}$$

where *W*(**Ω**) is a function of *λ*_1_, *λ*_2_, *θ*_1_, *θ*_2_and *π*_1_, *H*(**Ω**) is the logarithmic of joint prior for the parametric set **Ω**, and *K*(**Ω**|**x**) is the log-likelihood function, can be evaluated as

(16) $$\begin{array}{c} \begin{array}{c} I\left(\Omega \right)=W\left(\hat{\Omega }\right)+\left(\psi_{1}d_{1}+\psi_{2}d_{2}+\psi_{3}d_{3}+\psi_{4}d_{4}+\psi_{5}d_{5}+d_{6}+d_{7}\right)\\ +\frac{1}{2}\left(Q_{1}B_{1}+Q_{2}B_{2}+Q_{3}B_{3}+Q_{4}B_{4}+Q_{5}B_{5}\right), \end{array} \end{array}$$

where the MLE of **Ω** is denoted by$\hat{\Omega }$,

(17) $$\begin{array}{c} \begin{array}{c} B_{i}=\psi_{1}\omega_{i1}+\psi_{2}\omega_{i2}+\psi_{3}\omega_{i3}+\psi_{4}\omega_{i4}+\psi_{5}{\nu \omega }_{i5},\\ Q_{i}=\omega_{11}L_{11i}+\omega_{22}L_{22i}+\omega_{33}L_{33i}+\omega_{44}L_{44i}+\omega_{55}L_{55i}+2\omega_{12}L_{12i}+2\omega_{13}L_{13i}+2\omega_{14}L_{14i}+2\omega_{15}L_{15i},\\ +2\omega_{23}L_{23i}+2\omega_{24}L_{24i}+2\omega_{25}L_{25i}+2\omega_{34}L_{34i}+2\omega_{35}L_{35i}+2\omega_{45}L_{45i},\\ d_{i}=D_{1}\omega_{i1}+D_{2}\omega_{i2}+D_{3}\omega_{i3}+D_{4}\omega_{i4}+D_{5}\omega_{i5},i=1,2,3,4,5,\\ d_{6}=g_{12}\omega_{12}+g_{13}\omega_{13}+g_{14}\omega_{14}+g_{15}\omega_{15}+g_{23}\omega_{23}+g_{24}\omega_{24}+g_{25}\omega_{25}+g_{34}\omega_{34}+g_{35}\omega_{35}+g_{45}\omega_{45},\\ d_{7}=\frac{1}{2}\left(\psi_{11}\omega_{11}+\psi_{22}\omega_{22}+\psi_{33}\omega_{33}+\psi_{44}\omega_{44}+\psi_{55}\omega_{55}\right),\\ D_{i}=\frac{\partial H\left(\Omega \right)}{\partial \Omega_{i}},i=1,2,3,4,5,\Omega =\left(\lambda_{1},\lambda_{2},\theta_{1},\theta_{2},\pi_{1}\right)\xi_{ij}=\frac{\partial^{2}W\left(\Omega \right)}{\partial \Omega_{i}\partial \Omega_{j}},L_{ij}=\frac{\partial^{2}K\left(\Omega \left|x\right.\right)}{\partial \Omega_{i}\partial \Omega_{j}},i,j=1,2,3,4,5,\\ L_{ijv}=\frac{\partial^{3}K\left(\Omega \left|x\right.\right)}{\partial \Omega_{i}\partial \Omega_{j}\partial \Omega_{v}},i,j,v=1,2,3,4,5, \end{array} \end{array}$$

and *ω*_*ij*_ is the (*i*, *j*)^th^ element of the inverse of the matrix {*L*_*ij*_}.

Now, consider the log-likelihood function from (4).

(18) $$\begin{array}{c} \begin{array}{c} l\left(\Omega \left|x\right.\right)=\left(k_{1}+m_{1}\right)\log\pi_{1}+\left(k_{2}+m_{2}\right)\log\left(1-\pi_{1}\right)+\overset{2}{\underset{u=1}{\sum }}m_{u}\log\lambda_{u}+\overset{2}{\underset{u=1}{\sum }}m_{u}\log\theta_{u}\\ +\overset{2}{\underset{u=1}{\sum }}\left(\lambda_{u}-1\right)\overset{n_{u}}{\underset{i=k_{u}+1}{\sum }}\log\left(1-e^{-\theta_{u}x_{ui}}\right)-\overset{2}{\underset{u=1}{\sum }}\theta_{u}\overset{n_{u}}{\underset{i=k_{u}+1}{\sum }}x_{ui}+\lambda_{u}k_{u}\log\left(1-e^{-\theta_{u}x_{k+1}}\right). \end{array} \end{array}$$

Differentiating (18) with respect to models parameters and equating the results to zero, we have

(19) $$\begin{array}{c} \frac{\partial l\left(\Omega \left|x\right.\right)}{\partial \lambda_{u}}=\frac{m_{u}}{\lambda_{u}}+k_{u}\log\left(1-e^{-\theta_{u}x_{k+1}}\right)+\overset{n_{u}}{\underset{i=k_{u}+1}{\sum }}\log\left(1-e^{-\theta_{u}x_{ui}}\right)=0,u=1,2, \end{array}$$

(20) $$\begin{array}{c} \frac{\partial l\left(\Omega \left|x\right.\right)}{\partial \theta_{u}}=\frac{m_{u}}{\theta_{u}}+\frac{k_{u}\lambda_{u}x_{k+1}e^{-\theta_{u}x_{k+1}}}{1-e^{-\theta_{u}x_{k+1}}}-\overset{n_{u}}{\underset{i=k_{u}+1}{\sum }}x_{ui}+\left(\lambda_{u}-1\right)\overset{n_{u}}{\underset{i=k_{u}+1}{\sum }}\frac{x_{ui}e^{-\theta_{u}x_{ui}}}{1-e^{-\theta_{u}x_{ui}}}=0,u=1,2 \end{array}$$

(21) $$\begin{array}{c} \frac{\partial l\left(\Omega \left|x\right.\right)}{\partial \pi_{1}}=\frac{k_{1}+m_{1}}{\pi_{1}}-\frac{k_{2}+m_{2}}{1-\pi_{1}}=0. \end{array}$$

Here, the numerical solutions of (19) to (21) will provide MLE $\hat{\Omega }=\left({\hat{\lambda }}_{1},{\hat{\lambda }}_{2},{\hat{\theta }}_{1},{\hat{\theta }}_{2},{\hat{\pi }}_{1}\right)$ of **Ω**. Since, the higher-order derivative form (18) are straightforward, they have not been reported. The inverse of matrix {*L*_*ij*_}based on second order derivatives is

(22) $$\begin{array}{c} {\left\{L_{ij}\right\}}^{-1}=\left[\begin{array}{ccccc} \omega_{11} & \omega_{21} & \omega_{31} & \omega_{41} & \omega_{51}\\ \omega_{12} & \omega_{22} & \omega_{32} & \omega_{42} & \omega_{52}\\ \omega_{13} & \omega_{23} & \omega_{33} & \omega_{43} & \omega_{53}\\ \omega_{14} & \omega_{24} & \omega_{34} & \omega_{44} & \omega_{54}\\ \omega_{15} & \omega_{25} & \omega_{35} & \omega_{45} & \omega_{55} \end{array}\right]\text{ where }i,j=1,2,3,4,5. \end{array}$$

Now, the BEs for parameters of 2CMGEM using SELF are

(23) $$\begin{array}{c} \begin{array}{c} \Omega_{i,S}={\hat{\Omega }}_{i}+\frac{1}{2}\left(Q_{1}\nu_{1i}+Q_{2}\nu_{2i}+Q_{3}\nu_{3i}+Q_{4}\nu_{4i}+Q_{5}\nu_{5i}\right)+\overset{2}{\underset{u=1}{\sum }}\left(\frac{\mu_{u1}-1}{{\hat{\lambda }}_{u}}-\tau_{u1}\right)\sigma_{iu}\\ +\overset{2}{\underset{u=1}{\sum }}\left(\frac{\mu_{u2}-1}{{\hat{\theta }}_{u}}-\tau_{u2}\right)\sigma_{i\left(u+2\right)}+\left(\frac{\mu_{13}-1}{{\hat{\pi }}_{1}}-\frac{\tau_{13}-1}{1-{\hat{\pi }}_{1}}\right)\sigma_{i5}. \end{array} \end{array}$$

The BEs for the model parameters using LA under ELF are

(24) $$\begin{array}{c} \Omega_{i,E}={\left\{\begin{array}{c} {\overset{\wedge }{\Omega }}_{i}^{-1}+\frac{1}{2}\left(-{\overset{\wedge }{\Omega }}_{i}^{-2}\nu_{ii}+Q_{1}\nu_{1i}+Q_{2}\nu_{2i}+Q_{3}\nu_{3i}+Q_{4}\nu_{4i}+Q_{5}\nu_{5i}\right)\\ +\overset{2}{\underset{u=1}{\sum }}\left(\frac{\mu_{u1}-1}{{\overset{\wedge }{\lambda }}_{u}}-\tau_{u1}\right)\sigma_{iu}+\overset{2}{\underset{u=1}{\sum }}\left(\frac{\mu_{u2}-1}{{\overset{\wedge }{\theta }}_{u}}-\tau_{u2}\right)\sigma_{i\left(u+2\right)}\\ +\left(\frac{\mu_{13}-1}{{\overset{\wedge }{\pi }}_{1}}-\frac{\tau_{13}-1}{1-{\overset{\wedge }{\pi }}_{1}}\right)\sigma_{i5} \end{array}\right\}}^{-1}. \end{array}$$

#### 2.3.2. MCMC Method

This sub-subsection discusses the BE for parameters *λ*_1_, *λ*_2_, *θ*_1_, *θ*_2_, and *π*_1_ by employing MCMC technique. To implement MCMC procedure, we reformatted (9) as

(25) $$\begin{array}{c} \begin{array}{c} g\left(\Omega \left|x\right.\right)\propto \pi_{1}^{\gamma_{1}-1}{\left(1-\pi_{1}\right)}^{\psi_{2}-1}\overset{2}{\underset{u=1}{\prod }}\lambda_{u}^{\gamma_{3u}-1}\exp\left\{-\lambda_{u}\kappa_{1u}\left(x_{ui}\right)\right\}\theta_{u}^{\gamma_{4u}-1}\exp\left\{-\theta_{u}\kappa_{2u}\left(x_{ui}\right)\right\}\\ \times {\left(1-\exp\left(-\theta_{u}x_{k+1}\right)\right)}^{\lambda_{u}k_{u}}\exp\left\{-\overset{n_{u}}{\underset{i=k_{u}+1}{\sum }}\log\left(1-\exp\left(-\theta_{u}x_{ui}\right)\right)\right\}, \end{array} \end{array}$$

where *γ*_1_ = *k*_1_ + *m*_1_ + *μ*_1_, *γ*_2_ = *k*_2_ + *m*_2_ + *τ*_1_, *γ*_3*u*_ = *m*_*u*_ + *μ*_2*u*_, *γ*_4*u*_ = *m*_*u*_ + *μ*_3*u*_, *κ*_1*u*_(*x*_*ui*_) = *τ*_2*u*_ − ∑_*i*=*k*_*u*_+1_^*n*_*u*_^log(1 − exp(−*θ*_*u*_*x*_*ui*_)), and *κ*_2*u*_(*x*_*ui*_) = *τ*_3*u*_ + ∑_*i*=*r*_1_+1_^*n*_1_^*x*_1*i*_.

From (25), the posterior densities can be written as

(26) $$\begin{array}{c} f_{1}\left(\pi_{1}\left|x\right.\right)\propto \text{Beta}\left(\gamma_{1},\gamma_{2}\right),\\ f_{2}\left(\theta_{u}\left|x\right.\right)\propto \text{Gamma}\left(\gamma_{4u},\kappa_{2u}\left(x_{ui}\right)\right), \end{array}$$

*f*_3_(*λ*_*u*_|*θ*_*u*_, *x*) ∝ Gamma(*γ*_3*u*_, *κ*_1*u*_(*x*_*ui*_)), where Beta(.) and Gamma(.) represent bBeta and gamma distributions, respectively.

(27) $$\begin{array}{c} f_{4}\left(\lambda_{u},\theta_{u}\left|x\right.\right)\propto \overset{2}{\underset{u=1}{\prod }}{\left(1-\exp\left(-\theta_{u}x_{k+1}\right)\right)}^{\lambda_{u}k_{u}}\exp\left\{-\overset{n_{u}}{\underset{i=k_{u}+1}{\sum }}\log\left(1-\exp\left(-\theta_{u}x_{ui}\right)\right)\right\}. \end{array}$$

The samples from the posterior density can be obtained using the following algorithm.

Step-1:draw *π*_1_^(*z*)^, *θ*_*u*_^(*z*)^, and *λ*_*u*_^(*z*)^ from *f*_1_(*π*_1_|*x*), *f*_2_(*θ*_*u*_|*x*), and *f*_3_(*λ*_*u*_|*θ*_*u*_, *x*), respectively.

Step-2:replicate Step-2 *m* times to obtain (*π*_1_^(1)^, *λ*_1_^(1)^, *λ*_2_^(1)^, *θ*_1_^(1)^, *θ*_2_^(1)^) to (*π*_1_^(*m*)^, *λ*_1_^(*m*)^, *λ*_2_^(*m*)^, *θ*_1_^(*m*)^, *θ*_2_^(*m*)^) for *z* = 1, 2, ⋯, *m*.

The starting *m*_0_ number of samples has been discarded to minimize the impact of initial guess. The BEs for model parameters are computed using the rest of *m*_1_ = *m* − *m*_0_ number of samples.

The BEs under SELF using MCMC are

(28) $$\begin{array}{c} \pi_{1,S}=\frac{\sum_{z=1}^{m_{1}}\pi_{1}^{\left(z\right)}f_{1}\left(\pi_{1}^{\left(z\right)}\left|x\right.\right)f_{4}\left(\lambda_{u}^{\left(z\right)},\theta_{u}^{\left(z\right)}\left|x\right.\right)}{\sum_{z=1}^{m_{1}}f_{4}\left(\lambda_{u}^{\left(z\right)},\theta_{u}^{\left(z\right)}\left|x\right.\right)}, \end{array}$$

(29) $$\begin{array}{c} \lambda_{u,S}=\frac{\sum_{z=1}^{m_{1}}\lambda_{u}^{\left(z\right)}f_{3}\left(\lambda_{u}^{\left(z\right)}\left|\theta_{u}^{\left(z\right)},x\right.\right)f_{4}\left(\lambda_{u}^{\left(z\right)},\theta_{u}^{\left(z\right)}\left|x\right.\right)}{\sum_{z=1}^{m_{1}}f_{4}\left(\lambda_{u}^{\left(z\right)},\theta_{u}^{\left(z\right)}\left|x\right.\right)}.. \end{array}$$

The BEs under ELF using MCMC are

(30) $$\begin{array}{c} \pi_{1,E}={\left\{\frac{\sum_{z=1}^{m_{1}}\pi_{1}^{-1\left(z\right)}f_{1}\left(\pi_{1}^{\left(z\right)}\left|x\right.\right)f_{4}\left(\lambda_{u}^{\left(z\right)},\theta_{u}^{\left(z\right)}\left|x\right.\right)}{\sum_{z=1}^{m_{1}}f_{4}\left(\lambda_{u}^{\left(z\right)},\theta_{u}^{\left(z\right)}\left|x\right.\right)}\right\}}^{-1}, \end{array}$$

(31) $$\begin{array}{c} \lambda_{u,E}={\left\{\frac{\sum_{z=1}^{m_{1}}\lambda_{u}^{-1\left(z\right)}f_{3}\left(\lambda_{u}^{\left(z\right)}\left|\theta_{u}^{\left(z\right)},x\right.\right)f_{4}\left(\lambda_{u}^{\left(z\right)},\theta_{u}^{\left(z\right)}\left|x\right.\right)}{\sum_{z=1}^{m_{1}}f_{4}\left(\lambda_{u}^{\left(z\right)},\theta_{u}^{\left(z\right)}\left|x\right.\right)}\right\}}^{-1}.. \end{array}$$

## 3. Results and Discussions

In this section, we have generated the simulated datasets from 2CMGEM using different sample sizes, different censoring rates, different true parametric values, different hyperparameters and different mixing weights. As all these factors can have the impact on the estimation, we have considered different situations for each of these factors. As discussed by Momoli et al. [22], these datasets represent the real data from environmental studies and provide convenience by avoiding issues with empirical comparisons. Since censoring is major interest in this study, we have focused on the comparison of complete datasets with censored ones. Different estimation methods and two loss functions have been used in order to explore the best combination of estimation method and loss function in our case. The data from the 2CMGEM with LDL have been generated using the following steps.

- Step-1: generate a sample of size ‘*n*' from 2CMGEM
- Step-2: draw a uniformly distributed random number (*u*) for each observation generated in Step-1
- Step-3: when *u* ≤ *π*_1_, take observation from 1^st^ component, otherwise from 2^nd^ component of 2CMGEM
- Step-4: let LDL is *x*_*k*_
- Step-5: the observations falling below LDL are assumed to be censored from each component
- Step-6: the observations greater than or equal to LDL have been used for analysis

The corresponding results are given in Tables 1–5 and in Figures 1 and 2 given in the followings. The estimates under simulated samples were replicated 10,000 times, and average of the estimates has been reported. In addition, in case of the MCMC method, the estimates were replicated 11,000 times. The starting 1000 replications were not included in the estimation to remove the impact of choice of starting values for the estimation. The Mathematica and R software has been used for numerical computations.

Figure 1 shows the impact of change in sample size and censoring rates on the performance of the estimates. Panel (a1) reports the average of relative estimates (AREs) for parameter (*λ*_1_) using different sample sizes and under various estimation methods. Panel (a2) presents the amounts of mean square errors (MSEs) for the estimates of parameter (*λ*_1_). Similarly, AREs and MSEs for the parameter (*θ*_1_) can be seen in Panels (a1) and (a2), respectively. These figures elucidate that the estimates are converging to the true parametric values with increase in sample size. It is also evident from these panels (a1)–(a4) that amounts of MSEs tend to decrease with increase in the sample size. The results also advocated that the performance of the estimates using the MCMC method assuming ELF is superior as compared to their competitors. The results for the estimates of other model parameters also exhibited the similar trend, please see Table 1.

The detailed analysis of the impacts imposed by the increased censoring rate (on the estimates) is fundamental in environmental studies. For that purpose, the simulated data have been used to compare the results under different censoring rates with the case when no censoring occurs. It will provide an idea about how well our proposed estimators are capable of tackling the censoring scenarios. The right panel (c1 and c2) in Figure 1 shows these results. Panel (c1) elucidates the impact of censoring rates when sample size is 20, whereas panel (c2) presents the impacts of censoring rates when sample size is 200. The results in these panels (c1) and (c2) have been reported under MCMC method using ELF, as performance of these estimators was observed to be better than their counterparts. From these panels (c1 and c2), it can be assessed that when the sample is small (*n* = 20), the increased censoring rates tend to slightly inflate the MSEs for the estimates of the model parameters. However, for the sufficiently large sample size (*n* = 200), the MSEs for the estimates under complete data and under 30% censored data are very much comparative. Hence, the proposed estimators are efficient enough to deal with left censored environmental datasets.

The sensitivity of the proposed estimators with respect different values of hyperparameters, different mixing weights, and different true parametric values has been investigated in Figure 2. All the reported results are based on the MCMC method assuming ELF due to their supreme efficiency as compared to their competitors. The results have been compared on the basis of values of scaled MSEs (SMEs). The SMEs have been obtained by the ratio of MSEs to the corresponding true parametric values. The comparison of the estimates for complete data and 20% censored data has been considered. The left panel (a1 and a2) of the figure investigates the sensitivity of the estimates with respect to change in the hyperparameters. We have used three sets of the hyperparameters resulting in three different priors. The prior number one (*P*1) is the main prior which has been assumed for the overall analysis. This prior has been defined on the basis of prior means approach. Using prior means approach the hyperparameters in the prior are chosen in such a manner that the mean of resulting prior is approximately equal to the corresponding true parametric value. The other two priors (*P*2 and *P*3) have been specified so that the respective prior means have been changed (increased and decreased) by 20% from that of *P*1. In panels (a1) and (a2), the *x*-axis represents the combination of prior and censoring rate. For example, *P*1 (0%) means the results under prior one (*P*1) with no censoring and *P*1 (20%) denotes results under prior one (*P*1) with 20% censored samples. Panel (a1) elucidates that in case of complete data, the change in prior parameters has a very little affect on the performance of the estimates. On the other hand, for 20% censored samples, the change in prior parameters has resulted in slightly inflated SMSEs. However, when sample size is increased to 200, the estimates under all three priors are quite similar and censoring has very little impact on the efficiency of the estimates. The corresponding numerical results can be seen in Tables 2 and 3.

The central panel (*B*1 and *B*2) represents the affect of choice of various true parametric values on the estimates. Three different sets of true parametric values have been used to assess the impact of variant true parametric values on proposed estimators. The parametric sets used are as follows: *S*1: (*λ*_1_ = 0.5, *θ*_1_ = 1.2, *λ*_2_ = 0.75, *θ*_2_ = 1.5, *π*_1_ = 0.45); *S*2: (*λ*_1_ = 0.5, *θ*_1_ = 1.2, *λ*_2_ = 1.5, *θ*_2_ = 3, *π*_1_ = 0.45); and *S*3: (*λ*_1_ = 1, *θ*_1_ = 2.4, *λ*_2_ = 0.75, *θ*_2_ = 1.5, *π*_1_ = 0.45). The *x*-axis represents the combination of true parametric values and censoring rates. For example, *S*1 (0%) indicates the estimates for *S*1 with no censoring and *S*1 (20%) represents the results for *S*1 with 20% censored samples. Panels (b1) and (b2) show the results for sample size 20 and 200, respectively. For *n* = 20, some fluctuations in the amounts of SMSEs have been observed for different parametric sets. However, for *n* = 200, there is very little effect of various true parametric values can be seen. The corresponding numerical results have been placed in Table 4.

Keeping the values for the model parameters fixed, the impact of changing the mixing parameter has been presented in panels (c1) and (c2), respectively. The *x*-axis line denotes Pi1: *π*_1_ = 0.25 with no censoring; Pi2: *π*_1_ = 0.45 with no censoring; Pi3: *π*_1_ = 0.75 with no censoring; Pi4: *π*_1_ = 0.25 with 20% censoring; Pi5: *π*_1_ = 0.45 with 20% censoring; and Pi6: *π*_1_ = 0.75 with 20% censoring. For *n* = 20, the increase in value of the mixing parameter imposes a positive impact on the estimation of the model parameters from the first component of the mixture, without seriously affecting the estimation for the other component of the mixture. Interestingly, for *n* = 200, the choice of larger true values for the mixing parameter still produce the improved estimation for the first component of the mixture.

## 4. Real Examples

We have used two real environmental datasets with LDL for illustrating the applicability of the methods proposed. The first dataset contains ammonium (NH-4) concentration (mg/L) in precipitation observed at Olympic National Park, Hoh Ranger Station (WA14). This dataset has been reported by Aboueissa [34] and was collected during January, 2009 to December, 2011 on a weekly basis. We named it as dataset-1. The dataset contains high proportion (46 out of 102) of observations which are below LDL. The observations of the dataset are <0.006, <0.006, 0.006, 0.016, <0.006, 0.015, 0.023, 0.034, 0.022, 0.007, 0.021, 0.012, <0.006, 0.021, 0.015, 0.088, 0.058, <0.006, <0.006, <0.006, <0.006, 0.074, 0.011, 0.121, <0.006, 0.007, 0.007, 0.015, <0.006, <0.006, <0.006, <0.006, <0.006, <0.006, <0.006, <0.006, <0.006, <0.01, <0.01, <0.01, 0.042, <0.01, 0.013, <0.01, 0.028, <0.01, <0.01, <0.01, 0.049, 0.036, <0.01, 0.011, 0.019, 0.253, <0.018, <0.01, 0.014, 0.08, <0.01, 0.065, <0.01, <0.01, <0.01, <0.01, <0.01, <0.01, <0.008, <0.008, <0.008, <0.008, 0.009, <0.008, 0.017, 0.012, 0.02, 0.009, 0.014, 0.03, 0.06, 0.031, 0.024, 0.013, 0.059, 0.009, 0.017, 0.033, 0.052, 0.015, 0.019, <0.008, <0.008, <0.008, <0.008, 0.009, 0.013, 0.023, 0.036, <0.008, 0.012, 0.03, 0.022, and 0.008. Approximately, 45% of the observations have been below LDL. The average for the observations is 0.0316 with variance as 0.0015. The second dataset (dataset-2) has also been reported by Aboueissa [34]. This dataset is about the manganese concentrations (ppb) in groundwater collected from five wells. Since two LDL were used to obtain the dataset, 2-component mixture (2CM) can be used to model it. This dataset consist of twenty-five values with six observations falling below LDL. Hence, the data contains approximately 24% observation below the lower detection limit. The values of the dataset are <5, 12.1, 16.9, 21.6, <2, <5, 7.7, 53.6, 9.5, 45.9, <5, 5.3, 12.6, 106.3, 34.5, 6.3, 11.9, 10, <2, 77.2, 17.9, 22.7, 3.3, 8.4, and <2. The mean for the observations is 25.43 and variance is 752.96. The numerical results using dataset-1 and dataste-2 have been given in Tables 6–11 and in Figures 3 and 4. We have compared the proposed model (2CMGEM) with different mixture models available in literature to model the environmental datasets with LDL. These models include 2CM of normal models (2CMNM), 2CM of log-normal models (2CMLNM), 2CM of gamma models (2CMGM), and 2CM of log-gamma models (2CMLGM). By comparing fits of 2CMGEM with the models avaiable in literature, we have found the possibility and suitability of proposed model in modeling the left censored environmental datasets. The proposed MCMC methods have also been compared with the classical methods (MLE and EM algorithm) already used for estimating such datasets. The optimal number of components for the proposed mixture model have also been explored using different goodness-of-fit criteria and test statistics.

The graphs showing goodness-of-fit for different mixture models have been presented in Figure 3. From these graphs, it can easily be assessed that 2CMGEM is more representative as compared to other models for both datasets. In case of dataset-1, 2CMGEM seems to be the best model followed by 2CMNM and 2CMGM, while 2CMLNM and 2CMLGM did not provide good fits. On the other hand for dataset-2, again 2CMGEM provides the best fits followed by 2CMLNM and 2CMGM. Conversely, 2CMLGM and 2CMNM did not provided reasonable.

The results have been given in Table 7 and Table 10, respectively. The LRT assumes model with smaller number of components under null hypothesis. Hence, in the comparison of GEM and 2CMGEM, the GEM has been assumed under null hypothesis. While, for comparison on 2CMGEM with high-order mixtures, the model under null hypothesis is 2CMGEM. From the results, it can be seen that 2CMGEM is the best model for modeling each dataset.

The graphical comparison of fits under different estimation methods has been presented in Figure 4, while the numerical comparison has been given in Tables 8 and 11. Figure 4 reveals that the estimates under the MCMC method using ELF exhibited better discription data. However, the slight departure for some points can be due to the particular sample. The departure for the estimates under traditionally used MLE and EM methods are pronounced. The numerical results in Tables 8 and 11 further justified these findings. Hence, the proposed estimators are significantly better than the traditionally used estimators.

## 5. Conclusion

The study is aimed at exploring the improved estimation for the heterogeneous environmental datasets with LDL. The earlier studies considered classical analysis (MLEs and EM algorithm) of such datasets with some specific mixture models. We have proposed Bayesian analysis for modeling such data. The employment of 2CMGEM has also been proposed, and the optimality of the proposed model has been discussed. Our results revealed significant gains in efficiencies for the proposed estimators. In addition, the proposed estimators are quite insensitive with respect to LDL, true parametric values, hyperparametric values, and mixing weights. Hence, the proposed estimators are quite convincing alternative to those existing in the literature.

The current methodology can be extended to incorporate the variance analysis, invariant analysis, and covariance analysis. The future work can also be for the cases where the data is right or doubly censored.

## Figures and Tables

**Figure 1:** Parametric estimates using different sample sizes and censoring rates.

**Figure 2:** Sensitivity of the estimates with respect to priors, mixing parameter, true parametric values, and censoring rates.

**Figure 3:** Comparison of fits from different mixture models.

**Figure 4:** Comparison of fits for using different estimators.

**Table 1:** The amounts of AREs and MSEs for the model parameters using different estimation methods.

n	CR	Average relative estimates (AREs)					Mean square error (MSEs)				
		*λ*_1_ = 0.5	*θ*_1_ = 1.2	*λ*_2_ = 0.75	*θ*_2_ = 1.5	*π*_1_ = 0.45	*λ*_1_ = 0.50	*θ*_1_ = 1.2	*λ*_2_ = 0.75	*θ*_2_ = 1.5	*π*_1_ = 0.45
20	MLE	1.3192	1.1499	1.2417	1.2040	1.1795	0.0407	0.0559	0.0324	0.0608	0.0216
	EM	1.3149	1.1461	1.2377	1.2001	1.1757	0.0397	0.0538	0.0314	0.0588	0.0210
	SELF(LA)	1.3172	1.1395	1.2355	1.1957	1.1725	0.0400	0.0508	0.0304	0.0571	0.0212
	ELF(LA)	1.2852	1.1064	1.2028	1.1625	1.1408	0.0341	0.0378	0.0241	0.0453	0.0181
	SELF(MCMC)	1.3078	1.1208	1.2213	1.1791	1.1577	0.0305	0.0505	0.0272	0.0510	0.0162
	ELF(MCMC)	1.2674	1.1006	1.1909	1.1536	1.1307	0.0241	0.0371	0.0202	0.0378	0.0128

50	MLE	1.1898	1.0882	1.1456	1.1246	1.0949	0.0198	0.0279	0.0165	0.0345	0.0103
	EM	1.1846	1.0728	1.1353	1.1116	1.0837	0.0191	0.0240	0.0149	0.0311	0.0099
	SELF(LA)	1.1848	1.0718	1.1348	1.1109	1.0831	0.0190	0.0237	0.0148	0.0309	0.0099
	ELF(LA)	1.1602	1.0519	1.1125	1.0897	1.0621	0.0161	0.0190	0.0121	0.0254	0.0084
	SELF(MCMC)	1.1708	1.0545	1.1191	1.0943	1.0675	0.0121	0.0202	0.0111	0.0234	0.0063
	ELF(MCMC)	1.1438	1.0381	1.0973	1.0750	1.0477	0.0096	0.0161	0.0089	0.0186	0.0050

100	MLE	1.1035	1.0498	1.0829	1.0737	1.0401	0.0114	0.0177	0.0104	0.0253	0.0058
	EM	1.1026	1.0490	1.0821	1.0729	1.0393	0.0112	0.0173	0.0101	0.0248	0.0057
	SELF(LA)	1.1014	1.0462	1.0800	1.0704	1.0371	0.0111	0.0169	0.0099	0.0243	0.0056
	ELF(LA)	1.0764	1.0257	1.0572	1.0486	1.0156	0.0094	0.0138	0.0082	0.0201	0.0048
	SELF(MCMC)	1.0958	1.0376	1.0729	1.0625	1.0299	0.0064	0.0168	0.0082	0.0201	0.0033
	ELF(MCMC)	1.0728	1.0244	1.0547	1.0467	1.0135	0.0051	0.0135	0.0066	0.0161	0.0026

200	MLE	1.0387	1.0235	1.0371	1.0374	1.0305	0.0058	0.0087	0.0053	0.0140	0.0028
	EM	1.0363	1.0211	1.0347	1.0350	1.0281	0.0056	0.0084	0.0052	0.0135	0.0028
	SELF(LA)	1.0294	1.0178	1.0295	1.0307	1.0234	0.0055	0.0080	0.0050	0.0131	0.0027
	ELF(LA)	1.0206	1.0102	1.0213	1.0227	1.0154	0.0050	0.0072	0.0045	0.0118	0.0025
	SELF(MCMC)	1.0266	1.0123	1.0254	1.0258	1.0189	0.0026	0.0080	0.0039	0.0102	0.0013
	ELF(MCMC)	1.0130	1.0023	1.0135	1.0148	1.0076	0.0022	0.0070	0.0032	0.0084	0.0011

**Table 2:** Effect of different censoring rates on the estimation using the MCMC method and ELF.

CR	*n* = 20					*n* = 200				
	*λ*_1_ = 0.50	*θ*_1_ = 1.2	*λ*_2_ = 0.75	*θ*_2_ = 1.5	*π*_1_ = 0.45	*λ*_1_ = 0.50	*θ*_1_ = 1.2	*λ*_2_ = 0.75	*θ*_2_ = 1.5	*π*_1_ = 0.45
0%	0.0190	0.0271	0.0159	0.0298	0.0100	0.0018	0.0057	0.0026	0.0073	0.0009
5%	0.0205	0.0304	0.0172	0.0320	0.0108	0.0019	0.0059	0.0027	0.0076	0.0009
10%	0.0223	0.0332	0.0186	0.0350	0.0119	0.0021	0.0063	0.0030	0.0081	0.0010
11%	0.0228	0.0340	0.0190	0.0358	0.0120	0.0021	0.0063	0.0030	0.0081	0.0010
20%	0.0241	0.0361	0.0202	0.0378	0.0128	0.0022	0.0065	0.0032	0.0084	0.0011
30%	0.0253	0.0380	0.0213	0.0398	0.0134	0.0023	0.0068	0.0033	0.0087	0.0011

**Table 3:** Effect of mixing parameter on the estimation of model parameters using MCMC method and ELF.

*π*_1_	CR	*n* = 20					*n* = 200				
		*λ*_1_ = 0.50	*θ*_1_ = 1.2	*λ*_2_ = 0.75	*θ*_2_ = 1.5	*π*_1_	*λ*_1_ = 0.50	*θ*_1_ = 1.2	*λ*_2_ = 0.75	*θ*_2_ = 1.5	*π*_1_
0.25	0%	0.0363	0.0303	0.0239	0.0227	0.0253	0.0042	0.0056	0.0038	0.0054	0.0022
0.45	0%	0.0340	0.0281	0.0245	0.0230	0.0258	0.0041	0.0053	0.0039	0.0055	0.0022
0.75	0%	0.0324	0.0268	0.0256	0.0244	0.0260	0.0040	0.0051	0.0040	0.0057	0.0023
0.25	20%	0.0413	0.0336	0.0259	0.0247	0.0276	0.0047	0.0062	0.0041	0.0059	0.0024
0.45	20%	0.0382	0.0309	0.0269	0.0252	0.0284	0.0045	0.0058	0.0043	0.0060	0.0024
0.75	20%	0.0360	0.0291	0.0283	0.0270	0.0295	0.0043	0.0056	0.0044	0.0063	0.0025

**Table 4:** Effect of different true parametric values on the estimation using MCMC method and ELF.

PS	CR	*n* = 20					*n* = 200				
		*λ*_1_	*θ*_1_	*λ*_2_	*θ*_2_	*π*_1_ = 0.45	*λ*_1_	*θ*_1_	*λ*_2_	*θ*_2_	*π*_1_ = .45
*S*1	0%	0.0340	0.0281	0.0245	0.0230	0.0258	0.0041	0.0053	0.0039	0.0055	0.0022
*S*2	0%	0.0342	0.0276	0.0272	0.0253	0.0237	0.0041	0.0053	0.0043	0.0057	0.0021
*S*3	0%	0.0354	0.0310	0.0250	0.0227	0.0250	0.0042	0.0054	0.0040	0.0054	0.0021
*S*1	20%	0.0382	0.0309	0.0269	0.0252	0.0284	0.0045	0.0055	0.0043	0.0060	0.0024
*S*2	20%	0.0396	0.0310	0.0305	0.0284	0.0268	0.0046	0.0057	0.0049	0.0062	0.0023
*S*3	20%	0.0407	0.0348	0.0280	0.0254	0.0281	0.0047	0.0059	0.0045	0.0061	0.0024

**Table 5:** Effect of different hyper-parameters on the estimation using MCMC method and ELF.

PS	CR	*n* = 20					*n* = 200				
		*λ*_1_ = 0.50	*θ*_1_ = 1.2	*λ*_2_ = 0.75	*θ*_2_ = 1.5	*π*_1_ = 0.45	*λ*_1_ = 0.5	*θ*_1_ = 1.2	*λ*_2_ = 0.75	*θ*_2_ = 1.5	*π*_1_ = 0.45
*P*1	0%	0.03395	0.02814	0.02455	0.02303	0.02578	0.0041	0.0053	0.0039	0.0055	0.0022
*P*2	0%	0.03415	0.02827	0.02463	0.02311	0.02590	0.0041	0.0053	0.0039	0.0055	0.0022
*P*3	0%	0.03421	0.02833	0.02470	0.02313	0.02594	0.0041	0.0053	0.0039	0.0055	0.0022
*P*1	20%	0.03815	0.03088	0.02688	0.02523	0.02836	0.0045	0.0058	0.0043	0.0060	0.0024
*P*2	20%	0.03848	0.03105	0.02705	0.02537	0.02854	0.0045	0.0059	0.0043	0.0060	0.0024
*P*3	20%	0.03949	0.03171	0.02760	0.02592	0.02912	0.0046	0.0060	0.0044	0.0062	0.0025

**Table 6:** Comparison of different models based on various goodness-of-fit criteria using real dataset-1.

Model	AIC	BIC	KS statistic	KS P.Value
2CMGEM	-291.7208	-281.5940	0.0792	0.8740
2CMNM	-270.5970	-260.4703	0.0947	0.6971
2CMLNM	-107.2395	-97.1128	0.6972	2.20E-16
2CMGM	-269.6410	-259.5142	0.1077	0.5825
2CMLGM	-251.4048	-241.2780	0.1877	0.0387

**Table 7:** Selecting optimal components for generalized exponential mixture model using dataset-1.

Model	AIC	BIC	KS value	KS P.Value	LRT value	LRT P.Value
GEM	-277.535	-273.485	0.149	0.168	236.206	0.001
2CMGEM	-291.082	-280.955	0.079	0.874	Reference	Reference
3CMGEM	-285.688	-269.485	0.136	0.255	3.916	0.367
4CMGEM	-279.720	-257.441	0.168	0.084	4.302	0.467
5CMGEM	-273.680	-245.325	0.181	0.050	11.793	0.533

**Table 8:** Estimates of model parameters and goodness-of-fit statistics for 2CMGEM using dataset-1.

Estimation method	*π*_1_	*λ*_1_	*λ*_2_	*θ*_1_	*θ*_2_	AIC	BIC	KS value	KS P.Value
MLE	0.3140	2.381	8.286	27.551	179.155	-291.082	-280.955	0.079	0.874
EM	0.3157	2.392	8.310	27.496	181.599	-291.211	-281.084	0.074	0.916
SELF(LA)	0.3179	2.404	8.343	27.441	182.849	-291.271	-281.144	0.075	0.913
ELF(LA)	0.3264	2.416	8.385	26.728	182.947	-291.508	-281.381	0.071	0.942
SELF(MCMC)	0.3281	2.421	8.409	27.002	184.844	-291.521	-281.394	0.070	0.944
ELF(MCMC)	0.3370	2.432	8.450	27.276	192.047	-291.879	-281.752	0.060	0.988

**Table 9:** Comparison of different models based on various goodness-of-fit criteria using real dataset-2.

Model	AIC	BIC	KS statistic	KS P.Value
2CMGEM	163.5945	168.3167	0.0763	0.9295
2CMNM	181.5014	186.2236	0.2775	0.0474
2CMLNM	165.3600	170.0822	0.1410	0.7951
2CMGM	166.2773	170.9995	0.1825	0.4952
2CMLGM	169.6096	174.3318	0.2062	0.3863

**Table 10:** Selecting optimal components for generalized exponential mixture model using dataset-2.

Model	AIC	BIC	KS value	KS P.Value	LRT value	LRT P.Value
GEM	164.085	165.974	0.187	0.463	17.569	0.001
2CMGEM	163.595	168.317	0.076	0.930	Reference	Reference
3CMGEM	169.690	177.245	0.147	0.750	8.428	0.133
4CMGEM	175.832	186.221	0.197	0.400	2.488	0.833
5CMGEM	181.960	195.183	0.220	0.276	3.299	0.984

**Table 11:** Estimates of model parameters and goodness-of-fit statistics for 2CMGEM using dataset-2.

Estimation method	*π*_1_	*λ*_1_	*λ*_2_	*θ*_1_	*θ*_2_	AIC	BIC	KS value	KS P.Value
MLE	0.2554	8.8372	4.5844	0.0440	0.1796	163.595	168.317	0.123	0.905
EM	0.2466	8.2961	4.5118	0.0427	0.1648	163.826	168.548	0.114	0.941
Self(la)	0.2429	8.2081	4.4452	0.0423	0.1639	163.816	168.538	0.112	0.950
Elf(la)	0.2413	8.2045	4.4565	0.0431	0.1641	163.830	168.553	0.111	0.954
SELF(MCMC)	0.2412	8.1208	4.3904	0.0421	0.1644	163.771	168.493	0.106	0.968
ELF(MCMC)	0.2408	8.0702	4.4586	0.0421	0.1701	163.676	168.398	0.091	0.993

## Data Availability

Data used in the article in available in the article.

## Abbreviations

AIC: Akaike information criteria
ARE: Average of relative estimates
BIC: Bayesian information criteria
ELF: Entropy loss function
EM: Expectation-maximization
KS: Kolmogorov Smirnov
LA: Lindley's approximation
LE: Estimates using LA and ELF
LRT: Likelihood ratio test
LS: Estimates using LA and SELF
LDL: Lower detection limit
MCMC: Markov chain Monte Carlo
ME: Estimates using MCMC and ELF
MS: Estimates using MCMC and SELF
MLE: Maximum likelihood estimation
MSE: Mean square error
SELF: Squared error loss function
2CM: 2-component mixture
2CMGM: 2CM of gamma models
2CMGEM: 2CM of generalized exponential model
2CMLGM: 2CM of log-gamma models
2CMLNM: 2CM of log-normal models
2CMNM: 2CM of normal models.
